# Mechanism of Jujube (*Ziziphus jujuba* Mill.) Fruit in the Appetite Regulation Based on Network Pharmacology and Molecular Docking Method

**DOI:** 10.1155/2022/5070086

**Published:** 2022-04-10

**Authors:** Yu Zhu, Ju Huang, Tao Shen, Rensong Yue

**Affiliations:** Hospital of Chengdu University of Traditional Chinese Medicine, Chengdu 610072, China

## Abstract

**Objective:**

To investigate the mechanism of jujube (*Ziziphus jujuba* Mill.) in appetite regulation based on network pharmacology.

**Methods:**

The active components and action targets of jujube were retrieved through the TCMSP and TCMID databases. GeneCards, DisGeNet, Therapeutic Target Database, and OMIM were used to screen the related targets for appetite, appetite suppression, and appetite regulation, and the intersection target of the two was selected. A protein-protein interaction (PPI) network was constructed. Important protein nodes and subnets were predicted based on the cytoHubba plug-in, and the hub gene was screened. Additionally, GO and KEGG pathway analyses were performed to obtain potential biological processes and signaling pathways of key targets. And the active ingredient-target-action pathway diagram was constructed.

**Results:**

A total of 16 active components were screened from jujube, including 131 action targets related to appetite and appetite regulation. Three key targets (MAOA, MMP2, and HSPB1) were screened out by MCODE analysis. KEGG enrichment analysis was mainly enriched in neuroactive ligand-receptor interaction, serotonin-containing synapse, gap junction, cAMP signaling pathway, and dopaminergic synapse. Molecular docking results showed that the components coclaurine, (−)-catenin, (+)-stepholidine, berberine, cianidanol, coclaurine, and moupinamide in jujube had strong binding activity to the main targets (ESR1, ADRA2C, and MMP2).

**Conclusion:**

Based on network pharmacology, the appetite modulating effects of jujube on multiple components, targets, and channels were explored, and the main active components of jujube were predicted to act on multiple signaling pathways to regulate appetite. The molecular docking results showed that the components in jujube had strong binding activity to the main targets, which provided new ideas and methods to further investigate the mechanisms of appetite regulation by jujube.

## 1. Introduction

Hyperphagia is one of the most common and intractable symptoms in diabetic patients and is an important culprit in disrupting glucose homeostasis [1]. Studies have shown that recurrent blood glucose fluctuations are an independent risk factor for increased diabetic complications and cardiovascular mortality, and hyperphagia is a key driver of blood glucose drift and disease progression. The existing diabetes treatment drugs GLP-1 agonists can play a role in suppressing appetite in diabetic patients by inhibiting the appetite center and delaying gastric emptying [2, 3]. However, these drugs are expensive and can cause varying degrees of vomiting, headache, nasopharyngitis, and significant weight loss.

Fatty and sweet foods can trap the spleen and stomach, which will lead to spleen deficiency for a long time and eventually become diabetic, manifesting as easy hunger. Supplementing spleen deficiency and responding to the sweet nature of the spleen is one of the main tools in the clinical treatment of hyperphagia in diabetes in Chinese medicine [4, 5]. Spleen deficiency and overflow of Qi are the keys to the pathogenesis of hyperphagia in type 2 diabetes (T2DM), and the main treatment rule is to “conform to the preference of the sick, use sweet herbs to treat the spleen” [4]. Clinical practice has shown that large doses of jujube (*Ziziphus jujuba* Mill.) decoction can produce the symptoms of gastric fullness in patients and then achieve good results in appetite control without producing more obvious blood glucose fluctuations, but can also assist other glucose-lowering treatment options to maintain blood glucose homeostasis [4, 5]. Some basic studies suggest that jujube components have antioxidant [6], improving insulin resistance [7], inducing cancer cell apoptosis [8], inhibiting *α*-glucosidase activity [9], and sedative-hypnotic effects [10]. However, there is a relative lack of research on the pharmacological mechanisms of action of jujube on appetite regulation.

Network pharmacology is a research method that uses high-throughput screening in databases, network visualization, and data analysis techniques to reveal the complex biological network relationships among drugs, targets, and diseases and to analyze and predict the pharmacological mechanisms of drugs [11]. Molecular docking is a powerful tool for predicting the affinity and binding mode of proteins and ligands. For a given protein and ligand (protein, DNA/RNA, or small molecule), their binding mode and free energy of binding can be predicted to investigate their functions and mechanisms of action [12]. Virtual screening based on molecular docking methods has become one of the required processes for drug development against specific target proteins [12]. By constructing a database based on the main components of jujube and establishing a Chinese medicine target dataset through target prediction, then constructing a compound-target network, constructing a protein-protein interaction (PPI) network [13], performing gene ontology (GO) function enrichment analysis [14], and performing pathway-based enrichment analysis, we can explain the effects of jujube on appetite regulation at the molecular level by constructing a multidimensional network of Chinese medicine chemical composition-target of action-disease target-PPI network. By constructing a multidimensional network of Chinese herbal chemical constituents-targets-disease targets-PPI network, we can explain the effects of jujube on appetite regulation at the molecular level.

## 2. Materials and Methods

### 2.1. Composition of Jujube

The Chinese medicine name jujube was used to obtain drug composition information using the TCMSP (https://tcmspw.com/tcmsp.php) [15] database, TCMID (https://www.megabionet.org/tcmid/) [16] database, and other Chinese medicine composition databases, including the number of ingredients, molecular name, and molecular mass. The structures were imported into PubChem (https://pubchem.ncbi.nlm.nih.gov/) [17] for searching and normalization, supplementing their PubChem CID, and downloading the SDF structures.

### 2.2. Screening of Active Ingredients in Jujube

ADMET [18] is the absorption, distribution, metabolism, excretion, and toxicity of a drug. ADME is the study of drug metabolism kinetics and is commonly used in contemporary drug design and screening. In this study, we used the ADMET Descriptors module of Discovery Studio 2017R2 to predict the ADMET parameters of herbal ingredients, based on which human intestinal absorption (ADMET_Absorption_Level) and ADMET-Aqueous Solubility was used for the screening of the Chinese herbal ingredients. Compounds with ADMET_Absorption_Level 0, 1, 2 and ADMET_Solubility_Level 1, 2, 3, 4 were selected for inclusion in the study.

### 2.3. Prediction Screening of Target Proteins of Active Ingredients of Jujube

The predictive screening of the active ingredient target proteins of jujube was performed using the following two steps: the smile structures of the screened active ingredients were entered into DrugBank (https://go.drugbank.com/) [19], Therapeutic Target Database (https://db.idrblab.net/ttd/) [20], and Swiss Target Prediction platform (https://www.swisstargetprediction.ch/) [21] to predict the relevant targets of the active ingredients of the herbs and select “Homo sapiens” for the screening. The targets of “Homo sapiens” species were selected for screening, and a database of active ingredient targets of jujube ingredients was constructed.

The target prediction was carried out according to the method of Fu et al. [22], and all targets in the target database were scored by deep learning and a Bayesian network algorithm. The network topology parameters were calculated according to the scores, and the targets of the active ingredients of jujube were screened for subsequent research.

### 2.4. Disease Target Screening

The search term “Appetite Depressants/Appetite/Appetite Regulation” was set and the GeneCards database (https://www.GeneCards.org/) [23], the DisGeNet database (https://www.disgenet.org/) [24], the Therapeutic Target Database, and the OMIM database (https://www.omim.org) [25] were used to obtain the disease-related targets. The GeneCards database was applied to screen genes with a score greater than 2.3, and the DisGeNet database was queried for genes derived from the CTD (https://ctdbase.org/)-human [26] database. The OMIM and Therapeutic Target Database were applied to collect disease-associated genes. The data obtained from the four databases were merged to take the intersection, and the duplicate or invalid genes were removed to build the disease target database.

### 2.5. PPI Network Construction and Screening of Hub Genes

STRING database [27] is a database for searching known proteins and predicting protein-protein interactions, which contains 2031 species containing 9.6 million proteins and 138 million protein-protein interactions. We used the STRING database to construct a PPI network for the intersection of compounds and disease targets. The intersection was taken for the targets of the active ingredient of the compound and the disease targets. The intersection targets were uploaded to the STRING database (https://string-db.org/). The information of the constructed PPI network was imported into Cytoscape 3.8.2 software [28], based on the cytoHubba [29] plug-in topological algorithm to predict the important protein nodes and subnetworks in the network. And this study used DEGREE (Degree Correlation), MNC (Maximum Neighborhood Component), MCC (Maximal Clique Centrality), EPC (Edge Percolated Component), CLONESS (Closeness Centrality), and visualized hub gene. Cluster analysis was performed using the plug-in MCODE [30] to find gene clusters by using the correlation between proteins in the network, derive subnetworks, extract the differential genes contained in each gene cluster, and analyze the subnetworks. The main biological processes of the targets in the subnetworks are analyzed by finding gene clusters using correlations between proteins in the network, deriving subnetworks, and extracting the differential genes contained in each gene cluster.

### 2.6. Functional Enrichment and Disease Enrichment Analysis

GO functional annotation analysis is a common approach to perform large-scale functional enrichment studies of genes, including biological process (BP), molecular function (MF), and cellular component (CC). The Kyoto Encyclopedia of Genes and Genomes (KEGG) pathway is a widely used database for storing information about genomes, biological pathways, diseases, and drugs. The screened hub genes were imported into the DAVID 6.8 database (https://david.ncifcrf.gov/) [31], and the species selection “Homo sapiens” was used for GO analysis and KEGG pathway analysis (*P* < 0.05) to analyze the key targets involved in the relevant biological processes. Signaling pathways were analyzed and visualized using Cytoscape software.

### 2.7. Construction of “Active Ingredient-Potential Target-Action Pathway” Network

Cytoscape 3.8.2 software [28] was used to construct the “active ingredient-potential target-action pathway” network. The network consists of three parts, namely, active ingredients, target proteins, and pathways, to analyze and explore the multicomponent-multitarget-multipathway mechanism of Chinese medicine for the treatment of diseases.

### 2.8. Molecular Docking of Key Targets and Components

Molecular docking was performed using CDOCK in the Receptor-Ligand International module of the software Discovery Studio 2017 R2 [32] to precisely dock and analyze the key targets and the main components of Chinese medicine. The 3D structures of the small molecule compounds of the main active ingredients of traditional Chinese medicine were downloaded from PubChem (https://pubchem.ncbi.nlm.nih.gov/) according to their PubChem_ID numbers and imported into Discovery Studio 2017 R2. The high-resolution crystal structures of the targets were downloaded from the PDB [33] (https://www.rcsb.org/pdb/home/home.do) protein database, and the active sites of the proteins were centered on the active amino acid sites of the original ligand action labeled in the crystal structure itself, and the corresponding “active pockets” were constructed, so that the system searches for “active pockets” near the active site and finally locates the “active pocket” information to the target “active pocket.”

The parameters of the CDOCKER algorithm [34] module were set as follows: Pose Cluster Radius was set to 0.5, Random Conformations was set to 10, Orientations to Refine was set to 10, and the rest of the default parameters were kept unchanged. The process is shown in Figure 1.

## 3. Results

### 3.1. Screening of Active Compounds in Jujube

A total of 21 chemical components were obtained from the database collected for the jujube (DZ), with the main structural types being flavonoids, phenylpropanoids, alkaloids, terpenoids, etc. Chinese medicine contains a large number of chemical components, and the DS software was used to predict the ADMET parameters of the chemical components contained in the compound based on their chemical structures, which helps to find the possible active components quickly. Finally, a total of 16 active ingredients were screened, and the corresponding information about the screened active ingredients is detailed in Table 1.

### 3.2. Screening of Appetite-Related Targets in Jujube

The targets with *p* value >0.9 were screened from the prediction results of the target database as active ingredient targets, and a total of 194 active ingredient targets were obtained from the Chinese herbal compound. A larger number of targets were screened in the GeneCards database according to the search term “Appetite,” and 3330 targets were selected based on the criterion of score >2.3. 224 targets were obtained from OMIM database, and 275 targets were obtained from DisGeNEt. A total of 3552 targets were obtained after combining and deweighting, with 275 targets in OMIM database, 275 targets in DisGeNEt database, and 1 target in TTD database. The 194 potential targets of Chinese herbal ingredients were intersected with 3552 targets of disease targets, and a Wayne diagram was drawn (Figure 2(a)), and 131 potential targets of Chinese herbal compounds were initially obtained, and a compound name-Chinese herbal medicine-drug target interaction network was constructed (Figure 2(b)).

### 3.3. Construction of the PPI Network and Screening of Key Targets

The screened potential targets were input into the STRING database to obtain the target protein interaction information and imported into Cytoscape to construct the PPI network (Figure 3(a)), which had 130 nodes (target proteins) and 1004 edges (protein interactions). It indicated that among the predicted disease-related targets, the more targets could have effective interactions with that target. Using the five parameters of MNC, DEGREE, MCC, CLONESS, and EPC for screening (Figure 3(b)), the algorithm's computational analysis of the network structure and weighted linkage between nodes could screen out important key genes. The intersection of the top 30 results of each algorithm was taken to obtain 11 key targets (Figure 3(c), Tables 2 and 3).

### 3.4. Subnetwork Analysis

MCODE subnetwork analysis can discover more closely connected groups or genes in the network. It is calculated by weighting the points with the highest weight and set as SEED, from SEED, recursively move outward to find nodes that can join the subnetwork. Subnetwork 1 is centered on MAOA, and the important targets connected to it, such as SLC6A3, DRD3, DRD4, SLC18A2, and HTR1A, are all dopaminergic synapse-related targets, indicating that subnetwork 1 is closely related to dopaminergic synapses (Figure 4(a)). The core of subnetwork 2 is MMP2, and the important targets connected with it, such as TNF, are all targets related to inflammatory processes, indicating that subnetwork 2 is closely related to the regulation of tryptophan channels by inflammatory mediators (Figure 4(b)). The core of subnetwork 3 is HSPB1, and the important targets connected with it, such as CHRNA4, BRCA1, and HTR3A, are all targets related to cAMP signaling pathway, indicating that subnetwork 3 is closely related to cAMP signaling channels (Figure 4(c)).

### 3.5. GO Enrichment Analysis

In order to explore the functional distribution of key targets, 131 key targets were entered into the DAVID 6.8 database for GO enrichment analysis. The results showed 343 biological processes, 103 molecular functions, and 58 cellular components. Combined with the literature, the key targets in the biological process were filtered by *P* < 0.5 and the number of enriched targets was high, and the key targets were concentrated in response to stimulus, signaling, cell proliferation, positive regulation of biological process, negative regulation of biological process, etc. (Figure 5(a) and Table 4). Among the molecular functions, molecular transducer activity, catalytic activity, transporter activity, and transcriptional regulation activity are mainly involved (Figure 5(b) and Table 4). Among the cellular components, the membrane is the most involved target, followed by synapse, organelle part, and cell junctions (Figure 5(c) and Table 4).

### 3.6. KEGG Pathway Analysis

The KEGG pathway enrichment analysis of potential targets by the DAVID 6.8 data platform (*P* < 0.05) is shown in Figures 6(a)–6(d). The top 10 pathways were Neuroactive ligand-receptor interaction, Serotonergic synapse , Gap junction, cAMP signaling pathway, Dopaminergic synapse, Calcium signaling pathway, Hypoxia-inducible factor pathway (HIF-1 signaling pathway), Prolactin signaling pathway, Thyroid hormone signaling pathway, and Inflammatory mediator regulation of TRP channels (Table 5). It is suggested that jujube components may exert appetite modulating effects through the above pathways.

### 3.7. “Active Ingredient-Key Target-Pathway” Network Construction for Jujube

The active ingredients, potential targets, and selected signaling pathways of jujube were imported into Cytoscape 3.8.2 software to construct the “jujube-active-ingredient-target-action pathway” diagram (Figure 7(a)). The MCC algorithm of cytoHubba was used to further calculate the closest association of each component with key targets (Figure 7(b)). The results concluded that 5-hydroxytryptamine (5-HT)-containing synapses was the key pathway of action.

### 3.8. Molecular Docking Simulation of Target Interaction with Related Compounds

The docking of key target genes and their related compounds revealed that the docking binding energies of the targets and their related compounds were all negative (Table 6), indicating that the related compounds bind well to the targets. Among them, coclaurine had the lowest docking binding energy of −8.38 with ESR1, (−)-Catechin and ESR1, (+)-Stepholidine and ADRA2C, Berberine and ADRA2C, Cianidanol and ESR1, Coclaurine and ESR1, Moupinamide and MMP2, Quercetin and SCR, and Quercetin and TNF all had binding energies <−5 kcal/mol, and the binding patterns are shown in Figures 8(a)–8(h).

## 4. Discussion

Chinese medicine is difficult to elucidate molecular mechanisms due to the complexity of their chemical composition. Network pharmacology has been increasingly applied to the study of Chinese pharmaceutical preparations in recent years [11]. It transforms drug research from a “single target, single drug” model to a “network target, multicomponent therapy” model [35]. Studies have shown a favorable effect of jujube on glycosylated hemoglobin and some antioxidant effects in patients with T2DM [36]. However, for the time being, no studies have been conducted to analyze the network pharmacology of the active ingredients of jujube. Therefore, in this study, based on network pharmacology and molecular docking research methods, we constructed a multidimensional network through target prediction and protein interaction networks to elucidate the principle of action of jujube in treating diabetic hunger and regulating appetite from molecular prediction level.

In the present study, a total of 16 components including coclaurine, (−)-catenin, (+)-stepholidine, berberine, cianidanol, coclaurine, and moupinamide were identified as potential active ingredients of jujube. These active ingredients include 131 targets of action related to appetite and appetite regulation. Through PPI network analysis of jujube in appetite regulation, we identified 11 key targets: MAPK3, EGFR, SRC, HSP90AA1, and so on. For further screening by MCODE analysis, three key targets (MAOA, MMP2, and HSPB1) were identified. The molecular docking results showed that the main components of jujube had strong binding activity to the main targets (ESR1, ADRA2C, and MMP2).

MAOA can metabolize monoamine neurotransmitters [37]. Studies have shown that MAOA regulates food intake and energy expenditure [38]. Gardner et al. [39] similarly showed that MAOA is involved in regulating appetite and food intake related to obesity genes. HSP27 regulates actin dynamics and thus cell motility [40]. The inhibition of feeding by fibroblast growth factor (FGF)-1 is accompanied by the induction of HSP27 in periventricular astrocytes [41]. MMP2 is an endopeptidase that reduces the basement membrane around adipocytes, thus promoting the development of adipocyte hypertrophy [42]. Studies have shown high levels of MMP2 gene expression in patients with T2DM [43]. Previous studies suggested that the significant anorexigenic effect of estradiol in male rats would be related to ESR1 present in the lateral hypothalamic region [44]. The results of molecular docking suggested that coclaurine had the lowest docking binding energy with ESR1 at -8.38. And the stronger binding activity of coumestrol to ESR1 in jujube may be related to the estrogen-like effect of coumestrol. The accuracy of network prediction was reflected from the side.

Further, GO enrichment and KEGG pathway enrichment analysis showed that key genes act on signaling pathways such as neuroactive ligand-receptor interaction, serotonergic (5-hydroxytryptamine; 5-HT) synapse, cAMP signaling pathway, dopaminergic synapse, calcium signaling pathway, and hypoxia-inducible factor pathway. Among them, the key pathway of 5-HT synapses was closely related to appetite control and the treatment of related diseases. The key role of 5-HT in appetite control was formally proposed almost 30 years ago [45]. Studies have shown that the biogenic amine neurotransmitter 5-HT is negatively correlated with food intake and that a decrease in food intake is associated with 5-HT [46]. Agonists of 5-HT improve obesity and glycemic control in the population [47].

However, it should be noted that network pharmacology is based on existing databases and results for network modeling, and there is a certain false-positive rate of predicted results due to the differences in raw experimental data under different experimental conditions.

This paper presents a predictive analysis of the appetite regulation mechanism of jujube based on the theoretical level, and we hope that the results of this analysis can provide new ideas for the next in-depth research, and we also expect better research basis at the level of new drug development. Our research team will continue to focus on the progress of pharmacological research on jujube and will use the results of this paper as a reference to conduct relevant animal and cellular experiments to further investigate the effects and regulatory mechanisms of jujube on the appetite center of the hypothalamus.

## Figures and Tables

**Figure 1:** Flowchart.

**Figure 2:** Interaction network diagram of jujube for appetite treatment. (a) Venn diagram of jujube action targets and disease targets; (b) jujube-component-target interactions network. Green hexagon is Chinese medicine, red circle is component, and blue diamond is target.

**Figure 3:** Protein interaction network diagram. (a) All target protein interaction network; (b) top 30 target Venn diagram of MNC, DEGREE, MCC, CLONESS, and EPC; (c) key target protein interaction network diagram.

**Figure 4:** Subnetwork diagram. (a) Subnetwork 1; (b) subnetwork 2; (c) subnetwork 3. The larger the node, the darker the color means the higher the degree value of the target point.

**Figure 5:** GO enrichment analysis of the key targets. (a) Biological process (BP) analysis result; (b) molecular functions (MF) analysis result; (c) cellular components (CC) analysis result.

**Figure 6:** KEGG pathway enrichment results. (a) KEGG pathway network diagram; (b) KEGG enrichment pathway annotated classification results; (c) KEGG pathway enrichment circle diagram; (d) KEGG enrichment result bar graph.

**Figure 7:** Dates-component-target-pathway diagram. (a) Dazao-ingredient-target-pathway diagram; (b) the key target-ingredient diagram. The green hexagon is the name of a single herbal medicine, the red circle is the ingredient, the blue diamond is the target, and the purple arrow is the pathway name.

**Figure 8:** Molecular docking simulations of targets and compounds. (a) 3D and 2D plots of molecular docking of (−)-catechin-ESR1; (b) 3D and 2D plots of molecular docking of (+)-stepholidine-ADRA2C; (c) molecular docking 3D and 2D diagrams of berberine-ADRA2C; (d) molecular docking 3D and 2D diagrams of cianidanol-ESR1; (e) molecular docking 3D and 2D plots of coclaurine-ESR1; (f) molecular docking 3D and 2D plots of moupinamide-MMP2 target; (g) molecular docking 3D and 2D diagrams of quercetin-SCR; (h) molecular docking 3D and 2D diagrams of quercetin-TNF.

**Table 1:** Chemical composition and ADME parameters of jujube.

No.	Compound	PubChem CID	ADMET_Absorption_Level	ADMET_Solublity_Level	Herb
DZ1	(−)-Catechin	73160	0	3	Jujube
DZ2	(+)-Stepholidine	12442999	0	2	Jujube
DZ3	Berberine	2353	0	2	Jujube
DZ4	Betulinic acid	64971	2	1	Jujube
DZ5	Ceanothic acid	161352	2	1	Jujube
DZ6	Cianidanol	9064	0	3	Jujube
DZ7	Coclaurine	160487	0	3	Jujube
DZ8	Coumestrol	5281707	0	2	Jujube
DZ9	Malkangunin	90473155	0	3	Jujube
DZ10	Mauritine D	6443026	1	2	Jujube
DZ11	Moupinamide	5280537	0	3	Jujube
DZ12	Nuciferine	10146	0	2	Jujube
DZ13	Protopine	4970	0	2	Jujube
DZ14	Quercetin	5280343	1	3	Jujube
DZ15	Spiradine A	441756	0	3	Jujube
DZ16	Stepharine	98455	0	3	Jujube

**Table 2:** cytoHubba five-algorithm calculation results ranking.

Rank	MCC	CLONESS	MNC	EPC	DEGREE
1	MAOA	MAPK3	MAPK3	MAPK3	MAPK3
2	DRD2	EGFR	EGFR	SRC	EGFR
3	HTR1A	SRC	SRC	EGFR	SRC
4	DRD4	HSP90AA1	HSP90AA1	APP	HSP90AA1
5	DRD3	ESR1	TNF	HSP90AA1	TNF
6	SLC6A3	TNF	ESR1	ESR1	ESR1
7	SLC18A2	APP	APP	PIK3CA	APP
8	ADRA2C	PIK3CA	PIK3CA	TNF	PIK3CA
9	ADRA2A	BRCA1	BRCA1	RELA	BRCA1
10	HTR3A	RELA	GRIN2B	BRCA1	GRIN2B
11	HTR1B	GSK3B	SLC6A3	GSK3B	SLC6A3
12	CHRNA4	GRIN2B	HTR3A	GRIN2B	HTR3A
13	ACHE	MAPT	RELA	NTRK2	RELA
14	PIK3CA	PRKCA	CHRNA4	NFKB1	CHRNA4
15	HTR2A	PPARG	ACHE	CHRNA4	ACHE
16	ADRA1B	NTRK2	CDK1	DRD2	GSK3B
17	ADRA1A	NFKB1	DRD2	SLC6A3	CDK1
18	ADRA1D	CDK1	MAOA	PRKCA	DRD2
19	HTR2C	DRD2	NTRK2	ACHE	MAOA
20	HTR2B	ACHE	GSK3B	MAPT	PPARG
21	APP	HIF1A	PPARG	IGF1R	NTRK2
22	OXTR	CHRNA4	HIF1A	CDK1	HIF1A
23	F2	CDK5	MAPT	HIF1A	SLC18A2
24	NTSR1	GRIN1	MMP2	HTR3A	GRIN1
25	SRC	IGF1R	TOP2A	SLC18A2	MAPT
26	EGFR	ABCB1	NFKB1	PPARG	MMP2
27	MAPK3	PTPN1	SLC18A2	ADRA1B	TOP2A
28	HSP90AA1	MMP2	GRIN1	MAOA	NFKB1
29	ESR1	TOP2A	PRKCA	MCL1	PRKCA
30	RELA	F2	DRD4	GRIN1	DRD4

**Table 3:** Analysis of topological parameters of key targets.

Name	Closeness	Betweenness	Degree
ACHE	0.486792	0.014869	26
APP	0.565789	0.062058	39
CHRNA4	0.481343	0.011892	27
DRD2	0.490494	0.010911	26
EGFR	0.611374	0.077568	52
ESR1	0.570796	0.054579	42
HSP90AA1	0.586364	0.072456	46
MAPK3	0.641791	0.140011	58
PIK3CA	0.56087	0.052588	38
RELA	0.533058	0.011697	27
SRC	0.605634	0.073436	49

**Table 4:** GO analysis table.

Class	GO	Term	Count	*P* value
Molecular function	GO:0060089	Molecular transducer activity	54	2.19*E* − 24
	GO:0003824	Catalytic activity	74	4.44*E* − 09
	GO:0005215	Transporter activity	21	9.23*E* − 05
	GO:0005488	Binding	128	3.18*E* − 03
	GO:0104005	Hijacked molecular function	3	1.70*E* − 02
	GO:0016209	Antioxidant activity	3	2.42*E* − 02
	GO:0098772	Molecular function regulator	20	4.35*E* − 02
	GO:0140110	Transcription regulator activity	17	2.23*E* − 01
	GO:0005198	Structural molecule activity	4	7.77*E* − 01

Cellular component	GO:0045202	Synapse	49	5.58*E* − 23
	GO:0044456	Synapse part	34	3.96*E* − 15
	GO:0030054	Cell junction	30	2.44*E* − 08
	GO:0044425	Membrane part	81	4.76*E* − 08
	GO:0032991	Protein-containing complex	68	2.16*E* − 07
	GO:0016020	Membrane	96	6.75*E* − 07
	GO:0031974	Membrane-enclosed lumen	66	1.02*E* − 06
	GO:0044422	Organelle part	96	2.78*E* − 05
	GO:0005623	Cell	130	1.52*E* − 04
	GO:0044464	Cell part	130	1.52*E* − 04

Biological process	GO:0050896	Response to stimulus	125	3.86*E* − 29
	GO:0023052	Signaling	108	1.98*E* − 26
	GO:0032501	Multicellular organismal process	110	4.81*E* − 22
	GO:0048518	Positive regulation of biological process	99	5.94*E* − 21
	GO:0007610	Behavior	33	2.62*E* − 20
	GO:0008283	Cell proliferation	53	1.19*E* − 18
	GO:0048511	Rhythmic process	23	5.07*E* − 17
	GO:0048519	Negative regulation of biological process	88	5.95*E* − 17
	GO:0032502	Developmental process	91	4.46*E* − 15
	GO:0065007	Biological regulation	126	7.53*E* − 15

**Table 5:** KEGG pathway enrichment information.

Pathway	Count	*P* value
Neuroactive ligand-receptor interaction	30	1.28*E* − 15
Serotonergic synapse	18	4.07*E* − 14
Gap junction	15	3.49*E* − 12
cAMP signaling pathway	19	3.98*E* − 10
Dopaminergic synapse	14	1.04*E* − 08
Calcium signaling pathway	18	6.88*E* − 08
HIF-1 signaling pathway	10	9.55*E* − 06
Prolactin signaling pathway	8	1.60*E* − 05
Thyroid hormone signaling pathway	10	1.68*E* − 05
Inflammatory mediator regulation of TRP channels	9	1.73*E* − 05

**Table 6:** Molecular docking results of key targets and their related compounds.

Compound	Target	Combined energy (kcal/mol)
(−)-Catechin	ESR1	−7.01
	ADRA2C	−5.47

(+)-Stepholidine	ADRA2C	−7.10

Berberine	ADRA2C	−7.80

Cianidanol	ESR1	−7.14
	ADRA2C	−5.40

Coclaurine	ESR1	−7.02
	ADRA2C	−4.82

Coumestrol	ESR1	−8.38

Moupinamide	MMP2	−7.87
	EGFR	−4.03

Nuciferine	ADRA2C	−6.79

Quercetin	TNF	−7.61
	SRC	−6.95
	MMP2	−6.72
	MAPK3	−5.24
	HSP90AA1	−6.25
	ESR1	−7.36
	EGFR	−4.83
	APP	−4.57

## Data Availability

The data used to support the findings of this study are available from the corresponding author upon request.
